This article has been retracted.

# Expression Level and Clinical Significance of AK021443 in Non-Small-Cell Lung Carcinoma

**DOI:** 10.1155/2022/7957121

**Published:** 2022-03-14

**Authors:** Xiyong Wang, Yu Dai, Hongming Zhang, Honglin Xia, Qingsheng Kan

**Affiliations:** ^1^Department of Oncology, Suzhou Hospital Affiliated to Anhui Medical University (Suzhou Municipal Hospital), Suzhou, China; ^2^Department of Respiratory Medicine, Yancheng Third People's Hospital, The Affiliated Yancheng Hospital of Southeast University, Yancheng, China; ^3^Clinical Laboratory, Suzhou Hospital Affiliated to Anhui Medical University (Suzhou Municipal Hospital), Suzhou, China

## Abstract

To explore the prognostic potential of AK021443 in non-small-cell lung carcinoma (NSCLC), AK021443 levels in NSCLC specimens were determined by quantitative real-time polymerase chain reaction (qRT-PCR). The correlation between the AK021443 level and pathological factors in NSCLC patients was analyzed. Kaplan–Meier curves were plotted for assessing the prognostic value of AK021443 in NSCLC patients. Potential factors influencing NSCLC prognosis were analyzed by multivariable Cox regression test. AK021443 was upregulated in NSCLC specimens than normal ones. Its level was correlated to histological type, tumor differentiation, TNM staging, and lymphatic metastasis in NSCLC patients. AK021443 was the independent risk factor for the overall survival of NSCLC. AK021443 is highly expressed in NSCLC specimens, which is correlated to histological type, tumor differentiation, TNM staging, and lymphatic metastasis in NSCLC patients. It is the independent prognostic factor for NSCLC.

## 1. Introduction

Primary lung carcinoma is the most fatal tumor in the world. It is reported that, in 2015, up to 221,200 people were newly diagnosed as lung carcinoma, including 60% of deaths [1]. Usually, non-small-cell lung carcinoma (NSCLC) is the major histological subtype, accounting for over 80% of total lung carcinoma cases [2]. In the past decades, the average survival of NSCLC is shorter than 6 months [3]. With the improvement of living habits and changes in lifestyle and dietary, the incidence of NSCLC shows an annual increase [4]. At present, molecular biology technologies have been largely progressed. The therapeutic efficacy of NSCLC, however, is not optimistic [5, 6].

LncRNAs are a type of promising noncoding RNAs in medical research. They exceed 200 nt in length, and they are mainly distributed in the nucleus or cytoplasm. However, lncRNAs used to be interference signals in gene expressions [7]. Later, diverse biological functions of lncRNAs have been discovered, including their regulations on gene expression networks and signaling pathways [8]. LncRNAs can uniquely correlate with other nucleotides and proteins through complementary base pairing. Because of their regulatory effects, lncRNAs are extensively involved in pathological processes by mediating cell phenotypes and functions [9].

Very recently, abnormally expressed lncRNAs in NSCLC profiling have been identified, indicating that they may be novel biomarkers for NSCLC treatment [10]. MALAT1 is the first lncRNA used for molecular targeted therapy of lung carcinoma. Using antisense oligonucleotides (ASOs), knockdown of MALAT1 remarkably prevents NSCLC metastasis in mice [11]. Previous evidence [12] demonstrated that PVT1 is involved in NSCLC progression. Highly expressed PVT1 drives the deterioration of NSCLC. A recent study has proposed the prognostic potential of AK021443 in hepatocellular carcinoma [13]. So far, correlation analysis between AK021443 and NSCLC is rarely reported. In this paper, we aimed to analyze the clinical significance of AK021443 in NSCLC patients, which provides a novel biomarker for clinical treatment.

## 2. Materials and Methods

### 2.1. Baseline Characteristics of NSCLC Patients

A total of 200 NSCLC patients treated by radical resection were included. Histological subtypes and TNM staging in them were defined as previously reported [14, 15]. The inclusion criteria were as follows: (1) no limitation of gender; (2) clinical diagnosis of NSCLC; (3) no history of tumor; (4) no previous history of anticancer treatment; (5) reliable and detailed treatment file. The exclusion criteria were as follows: (1) clinically diagnosed as SCLC; (2) combined with other tumors; (3) loss of follow-up; (4) radical resection was not performed. The study was approved by the ethics committee of Suzhou Municipal Hospital. Written informed consent was obtained from each subject.

### 2.2. Follow-Up

Follow-up was conducted every three months in the first two years and every six months in the following three years. Overall survival (OS) was the primary endpoint, which was defined as the duration from the date of diagnosis to the date of death caused by any reason. For subjects who have been lost to follow-up before death, the time of the last follow-up was calculated as the time of death.

### 2.3. Quantitative Real-Time Polymerase Chain Reaction (qRT-PCR)

RNAs were isolated from blood samples of NSCLC patients using the commercial RNA isolation kit (TIANGEN Biotech, Beijing, China) and reversely transcribed to cDNAs (Applied Biosystems, Foster City, CA, USA). Amplification conditions were as follows: 95°C at 5 min and 35 cycles at 95°C for 10 s, 60°C for 30 s, and 72°C for 30 s. Primer sequences were as follows: AK021443, F: 5′-CTTGAACCCAGAAGACAGG-3′, R: 5′-ATGGAACATTAGAGGTAGCAC-3′; GAPDH, F: 5′-CGGATTTGGTCGTATTGGG-3′, R: 5′-GATTTTGGAGGGATCTCGC-3′.

### 2.4. Statistical Analyses

Statistical analyses were conducted by Statistical Product and Service Solutions (SPSS) 19.0 (IBM, Armonk, NY, USA). All data were expressed as mean ± SD (standard deviation). The *t*-test was used to compare the differences between two groups, and the chi-square test was used for the enumeration data. The correlation between the AK021443 level and pathological factors in NSCLC patients was analyzed by chi-square test. Kaplan–Meier curves were plotted for survival analysis. Potential factors influencing NSCLC prognosis were analyzed by multivariable Cox regression test. *P* < 0.05 was statistically significant.

## 3. Results

### 3.1. Upregulation of AK021443 in NSCLC

Two hundred cases of NSCLC specimens and paired normal ones were collected. qRT-PCR data showed a higher level of AK021443 in NSCLC specimens than controls (Figure 1(a)). We conducted as long as 5-year postoperative follow-up of each subject. Kaplan–Meier curves uncovered poor prognosis in NSCLC patients overexpressing AK021443 (HR = 14.65, *P* < 0.001) (Figure 1(b)). It is suggested that AK021443 was unfavorable to the prognosis in NSCLC.

### 3.2. Correlation between AK021443 and Pathological Factors in NSCLC

Recruited NSCLC patients were divided into two groups (*n* = 100) based on the median level of AK021443 in cancer specimens. As chi-square analysis demonstrated, AK021443 level was unrelated to age and gender in NSCLC patients (*P* > 0.05). According to the histological subtypes, the expression of AK021443 was significantly higher in lung adenocarcinoma than that in squamous cell carcinoma (*P* < 0.05). NSCLC patients with a high level of differentiation or advanced TNM staging had a higher level of AK021443 (*P* < 0.05). In addition, NSCLC patients with lymphatic metastasis expressed a higher level of AK021443 compared with nonmetastatic patients (*P* < 0.05) (Table 1). It is concluded that AK021443 was linked to histological subtype, tumor differentiation, TNM staging, and lymphatic metastasis in NSCLC patients.

### 3.3. Prognostic Factors of NSCLC

According to the conclusion obtained from the chi-square test, the four variables with significant differences (histological subtype, tumor differentiation, TNM staging, and lymphatic metastasis) and AK021443 were subjected to the Cox regression model. Potential factors influencing OS in NSCLC were assessed. It is found that tumor differentiation, TNM staging, and AK021443 level were independent factors predicting OS in NSCLC (*P* < 0.05) (Table 2).

### 3.4. Subgroup Analyses on Potential Factors Influencing OS in NSCLC

To further explore the prognostic potentials of AK021443 in NSCLC, we conducted subgroup analyses. In poorly differentiated NSCLC patients, AK021443 level was unrelated to OS (HR = 0.0889, *P*=0.7656) (Figure 2(a)). However, in well-differentiated NSCLC patients, OS was remarkably lower in those expressing a high level of AK021443 (HR = 3.910, *P*=0.048) (Figure 2(b)). AK021443 level was unrelated to OS in stage I + II NSCLC patients (HR = 2.290, *P*=0.1302) (Figure 2(c)), while it predicted poor OS in stage III + IV NSCLC patients with a high level of AK021443 (HR = 5.389, *P*=0.0203) (Figure 2(d)). In addition, no remarkable correlation between the AK021443 level and OS was identified in nonmetastatic NSCLC patients (HR = 0.8971, *P*=0.3436) (Figure 2(e)), while a high level of AK021443 predicted poor OS in NSCLC patients with lymphatic metastasis (HR = 11.06, *P* < 0.001) (Figure 2(f)). It is concluded that OS in NSCLC patients was linked to AK021443 level, tumor differentiation, TNM staging, and lymphatic metastasis.

## 4. Discussion

Comprehensive strategies, including surgery, chemotherapy, and radiotherapy, are preferred to NSCLC. The prognosis of NSCLC is extremely poor even though great efforts have been made on improving therapeutic efficacy [16–18]. A large proportion of NSCLC patients are diagnosed in the advanced stage of NSCLC, and 80% of them cannot be operated because of developed distant metastases [19]. It is urgent to seek for molecular biomarkers for early diagnosis and treatment guidance.

LncRNAs are widely involved in various aspects during tumor progression [20]. Multiple lncRNAs have been identified as oncogenic molecules triggering the malignant progression of NSCLC [21]. It is reported that overexpressed CCAT2 is only detected in adenocarcinoma of lung tissues, while it can hardly be detected in squamous cell carcinoma of lung tissues [22]. Meanwhile, a higher level of CCAT2 predicts worse prognosis in SCLC [23]. Nakagawa et al. [24] pointed out that the median survival is lower in NSCLC patients overexpressing HOTAIR [24]. Therefore, HOTAIR is considered as a promising biomarker for predicting prognosis in NSCLC. Long noncoding RNA AK021443 was reported to be related to some types of cancers; however, to date, no evidence reported AK021443 in lung cancer. Yang et al. showed that AK021443 may play an important role in tumorigenesis and progression and would be a powerful marker to predict the prognosis of hepatocellular carcinoma patients.

In this paper, we detected upregulated AK021443 in NSCLC specimens. A previous study has illustrated that knockdown of AK021443 obviously attenuates *in vivo* growth of hepatocellular carcinoma, and AK021443 is believed as a potential therapeutic target [25]. The novelty of the present study was that this is the first attempt to explore the role of AK021443 in lung cancer. Our findings showed that AK021443 level was linked to histological subtype, differentiation level, TNM staging, and lymphatic metastasis in NSCLC. In addition, OS in NSCLC patients was linked to AK021443 level, tumor differentiation, TNM staging, and lymphatic metastasis. To sum up, AK021443 has potential clinical significance in evaluating the prognosis of NSCLC, especially patients with unfavorable factors to the prognosis. Our study provides a new molecular marker for the clinical treatment and prognosis assessment of NSCLC.

Limitations still existed in the present study. We only investigated the potential role of AK021443 via analyses based on the clinical samples. Further exploration in lung cell lines and animal models should also be performed to elucidate the exact biofunctions of AK021443 in regulating the tumorigenesis of NSCLC and to study the underlying molecular mechanism in this biological process.

## 5. Conclusions

AK021443 is highly expressed in NSCLC specimens, which is correlated to histological type, tumor differentiation, TNM staging, and lymphatic metastasis in NSCLC patients. It is the independent prognostic factor for NSCLC.

## Figures and Tables

**Figure 1:** Upregulation of AK021443 in NSCLC. (a) AK021443 level in NSCLC specimens and normal ones. (b) Overall survival in NSCLC patients based on the AK021443 level (HR = 14.65, *P* < 0.001).

**Figure 2:** Subgroup analyses on potential factors influencing OS in NSCLC. (a, b) Overall survival in poorly differentiated (a) or well-differentiated NSCLC patients (b). (c, d) Overall survival in stage I + II (c) or stage III + IV NSCLC patients (d). (e, f) Overall survival in lymphatic metastatic (e) or nonmetastatic NSCLC patients (f).

**Table 1:** Correlation between the AK021443 level and pathological factors in patients with non-small-cell lung carcinoma.

Variable	*n*	Low level (*n* = 100)	High level (*n* = 100)	*χ* ^2^	*P*
*Sex*					
Male	128	61	67	0.791	0.462
Female	72	39	33		
*Age*					
<60	81	37	44	1.017	0.194
≥60	119	63	56		
*Histological type*					
Adenocarcinoma	111	37	74	27.715	<0.001
Squamous cell carcinoma	89	63	26		
*Differentiation*					
Poorly	95	60	35	12.531	0.001
Well	105	40	65		
*TNM staging*					
I + II	84	54	30	11.823	0.001
III + IV	116	46	70		
*Lymphatic metastasis*					
No	74	50	24	14.5	<0.001
Yes	126	50	76		

**Table 2:** Potential factors influencing NSCLC prognosis analyzed by multivariable Cox regression test.

Variables	HR	95% CI	*P*
Differentiation (poorly vs. well)	2.761	1.879–4.335	0.027
TNM staging (I + II vs. III + IV)	1.893	1.243–2.682	<0.001
Lymphatic metastasis (no vs. yes)	1.769	0.783–3.214	0.086
AK021443 level (low vs. high)	2.538	1.763–3.559	0.004

HR: hazard ratio; CI: confidence interval.

## Data Availability

The datasets used and analyzed during the current study are available from the corresponding author upon reasonable request.
